# Machine Learning for Predicting Hyperglycemic Cases Induced by PD-1/PD-L1 Inhibitors

**DOI:** 10.1155/2022/6278854

**Published:** 2022-08-19

**Authors:** Jincheng Yang, Ning Li, Weilong Lin, Liming Shi, Ming Deng, Qin Tong, Wenjing Yang

**Affiliations:** ^1^Office for Cancer Diagnosis and Treatment Quality Control, National Cancer Center, National Clinical Research Center for Cancer, Cancer Hospital, Chinese Academy of Medical Sciences and Peking Union Medical College, Beijing, China; ^2^Department of Comprehensive Oncology, National Cancer Center, National Clinical Research Center for Cancer, Cancer Hospital, Chinese Academy of Medical Sciences and Peking Union Medical College, Beijing, China; ^3^Department of Acupuncture and Moxibustion, Wuhan Xinzhou District Hospital of Traditional Chinese Medicine, Wuhan, Hubei, China

## Abstract

**Objective:**

Immune checkpoint inhibitors, such as programmed death-1/ligand-1 (PD-1/L1), exhibited autoimmune-like disorders, and hyperglycemia was on the top of grade 3 or higher immune-related adverse events. Machine learning is a model from past data for future data prediction. From post-marketing monitoring, we aimed to construct a machine learning algorithm to efficiently and rapidly predict hyperglycemic adverse reaction in patients using PD-1/L1 inhibitors.

**Methods:**

In original data downloaded from Food and Drug Administration Adverse Event Reporting System (US FAERS), a multivariate pattern classification of support vector machine (SVM) was used to construct a classifier to separate adverse hyperglycemic reaction patients. With correct core SVM function, a 10-fold 3-time cross validation optimized parameter value composition in model setup with R language software.

**Results:**

The SVM prediction model was set up from the number type/number optimization method, as well as the kernel and type of “rbf” and “nu-regression” composition. Two key values (nu and gamma) and case number displayed high adjusted *r*^2^ in curve regressions (*nu* = 0.5649 × *e*^(− (case/6984))^, gamma = 9.005 × 10^−4^ × case − 4.877 × 10^−8^ × case^2^). This SVM model with computable parameters greatly improved the assessing indexes (accuracy, F1 score, and kappa) as well as coequal sensitivity and the area under the curve (AUC).

**Conclusion:**

We constructed an effective machine learning model based on compositions of exact kernels and computable parameters; the SVM prediction model can noninvasively and precisely predict hyperglycemic adverse drug reaction (ADR) in patients treated with PD-1/L1 inhibitors, which could greatly help clinical practitioners to identify high-risk patients and perform preventive measurements in time. Besides, this model setup process provided an analytic conception for promotion to other ADR prediction, such ADR information is vital for outcome improvement by identifying high-risk patients, and this machine learning algorithm can eventually add value to clinical decision making.

## 1. Introduction

Diabetes mellitus and cancer are among the leading causes of death worldwide. As a major contributor to neoplastic transformation and an important prediabetes index, hyperglycemia (high blood glucose) is also influenced by cancer treatment. Higher blood glucose level, dealing with or without insulin, may lead to serious complications of diabetes, such as ketoacidosis, and is correlated with cancer risk, progression, and mortality at a higher degree [1–3].

Recently, immunotherapy is a vast improvement among anticancer therapies [4]. In 2018 and 2019, JAMA Oncology reported treatment-related adverse events from programmed death-1 (PD-1) inhibitors, programmed death ligand-1 (PD-L1) inhibitors, and immune checkpoint inhibitor regimens in clinical trials. Among the endocrine dysfunctions, hyperglycemia was the third (after hypothyroidism and hyperthyroidism) at all-grade immune-related adverse events (irAEs) and the first at grade III or higher irAEs [5, 6]. Our previous research indicated that Nivolumab and Pembrolizumab were positive hyperglycemia-causing drugs [7, 8]. In 2021, JAMA Oncology reported that risks of chronic irAEs should be integrated into treatment decision making [3]. Prolonged exposure to hyperglycemia can epigenetically modify gene expression profiles in human cells, and this effect is sustained even after blood glucose is therapeutically controlled. Cancer cells exposed to hyperglycemia would grow permanently and aggressively, even after euglycemia returned. This metabolic phenomenon is called hyperglycemic memory, which contributes substantially to the pathology of various diabetic complications [9, 10].

Worldwide public database on adverse events could provide many drug-usage information [11, 12], having become a new information source in drug post-marketing phase. US Food and Drug Administration (FDA) is responsible for protecting the public health by ensuring the safety, efficacy, and security of drugs, biological products, and medical devices. The reports of Food and Drug Administration Adverse Event Reporting System (FAERS) are evaluated by clinical reviewers to monitor the safety of products after they are approved. FAERS is such a database that contains adverse event reports, medication error reports, and product quality complaints resulting in adverse events. The database is designed to support the FDA's post-marketing safety surveillance program for drug and therapeutic biologic products. The informatic structure of the FAERS database adheres to the international safety reporting guidance issued by the International Conference on Harmonization [13].

Machine learning (ML) “learns” a model from past data in order to predict future data. The key process is the learning which is one of the artificial intelligences [14]. Artificial intelligence-based solutions can improve medication safety with minimal overhead for patients and health professionals [15]. Machine learning focuses on how computers learn from data, using its emphasis on efficient computing algorithms [16, 17]. In health record field, machine learning techniques have been a hot spot in data mining; trajectory data mining has become an important research direction [18]. Modeling this big data information requires managing overfitting, model interpretability, and computational cost [19]. It offers a lot of advantages for assimilation and assessment of complex health big data, including flexibility and scalability, which is widely used in risk stratification, diagnosis, classification, and survival predictions. Health data's diversity trait calls for machine learning at demographic records, laboratory findings, images, or doctors' records, as well as predictions for disease risk, diagnosis, prognosis, and appropriate treatments [20].

Many different statistical, probabilistic, and optimization techniques can be implemented as learning methods such as the logistic regression, artificial neural networks, K-nearest neighbor, decision trees, and Naïve Bayes [14]. However, traditional biostatistical methods (e.g., logistic regression or linear regression) could not provide higher precision in health-data prediction, especially in real-world research. Support vector machine (SVM) is widely used as a type of supervised learning algorithm which analyzes data and recognizes patterns, mainly used for binary classification and regression by linear or nonlinear decision boundary [21]. It aims to divide samples into worthy bifurcations that enable the prediction of labels from one or more feature vectors. This decision boundary, through a line or plane called the maximum margin hyperplane in multidimensional feature, is orientated in such a way that it is as far as possible from the closest data points from each of the classes. These closest points are called support vectors. SVM is powerful at recognizing subtle patterns in complex datasets, being used to recognize handwriting, recognize fraudulent credit cards, and identify a speaker, as well as detect face [14].

SVM-based approach performances well in managing sparse data in high dimensions, in that it overcomes the other state-of-the-art competitors providing the best compromise between prediction and computation time [19]. It has been applied to seizure prediction, detection, and classification [22]. One advantage of SVM is its classification of small number of training samples; another is solving linear and nonlinear regression problems [23].

To date, the correlation of hyperglycemic occurrences and personal-related features, or which kinds of special features could mostly correlate with hyperglycemia, has become an urgent problem, for which all of these predictions have not been reported yet. Predicting and avoiding terrible ADR can provide better guidance for clinical decision making. In this study, we aimed to construct an effective SVM-based machine learning model with high accuracy, low computational costs, and computable parameters to predict hyperglycemia in PD-1/PD-L1–treated patients.

## 2. Methods

### 2.1. Data Sources

Original data was downloaded from US FAERS public dashboard [13] (data retrieval date: Dec 31, 2021).

#### 2.1.1. Inclusion Criteria

Inclusion criteria were as follows:

- Drugs: Camrelizumab (cam, PD-1), Cemiplimab (cem, PD-1), Avelumab (avel, PD-L1), Durvalumab (dur, PD-L1), Atezolizumab (atez, PD-L1), Pembrolizumab (pem, PD-1), Nivolumab (nivo, PD-1), and Ipilimumab (ipi, CTLA-4).
- Positive cases: Items in “Reaction” variable including at least one of the following: “Diabetes Mellitus,” “Diabetic,” “Hyperglycaemia,” “Hyperglycinaemia,” “Glucose Tolerance Impaired,” and “Blood Glucose Increased.”

#### 2.1.2. Exclusion Criteria

Exclusion criteria were as follows:

- Cases with wrong report year.
- Variables with no healthcare information (Step 1.1).
- Cases with missing value(s), excluded in complete data (Step 1.2).

### 2.2. Procedure

The procedure comprises data download, algorithm selection, key parameter regression, and model prediction performance (Figure 1).

Step 1. Data Version
    Step 1.1. Variable primary screening
    Variables (13 columns) were obtained from the downloaded Excel files: Case ID, Reason for Use, Reactions, Serious, Outcomes, Sex, Event Date, Case Priority, Patient Age, Patient Weight, Reporter Type, Report Source, and Country where event occurred.
    Variables (11 columns) with no more healthcare information were excluded: Suspected Product Names, Suspected Product Active Ingredients, Latest FDA Received Date, Sender, Concomitant Product Names, Latest Manufacturer Received Date, Initial FDA Received Date, Reported to Manufacturer, Manufacturer Control Number, Literature Reference, and Compounded Flag.
    Step 1.2. Raw data and complete data
    Original data were fixed into two versions: raw data (cases with missing values) and complete data (deleted cases with missing value(s)). The two versions of data contained above 13 variables.
Step 2. Core SVM algorithm
Positive and negative cases could be substituted as 2-category factor type (“Yes” and “No”) or number type (“1” and “0”) in SVM model setup.
There are two parameter optimization methods: number optimization and *R*-function optimization. In number optimization, the best values were defined by the composition of parameters, according to the best range of each parameter. In *R*-function optimization, the parameter range was input to a built-in function (*R* library: tune.svm). If the best values were close to range boundary, the new range would be adjusted for optimization again. The factorized data were optimized via both number and function methods.
    Step 2.1. Number/factor
    Each drug with 600 cases (positive and negative cases proportionally) was extracted from raw data and complete data. All the type-optimization compositions were tested. In raw data, the results of factor number were very close to those of factor tune, so they are only displayed as “*f*_raw” and “*n*_raw.” As *R*-tune optimization needs variables in form of factor, there were no results of “nr” (number type/*R*-tune optimization), but only “*nn*” (number type/number optimization).
    The data version was also determined at this step.
    Step 2.2. Variables
    The key to construct an SVM model that can screen the active markers accurately is to select the appropriate variables. Variable selection was according to two methods: near zero variance method (*R* library: nearZeroVar; “*T*” means deletable) and model assessment (R library: varImp; “0” means deletable).
    Step 2.3. Type and kernel
    Parameter selection: parameters from *R* language library SVM (e1071) official Arguments are as follows: SVM-Type (*C*-classification, “*C*”; one-classification, “one”; eps-regression, “eps”; nu-regression, “nu”) and SVM-Kernel (linear, “*l*”; poly, “*p*”; radial basis (rbf), “*r*”; sigmoid, “*s*”).
    Selection is also based on data types (number and factor). “eps” and “nu” regression need numeric dependent variables, while “one” and “*C*” classification can accept both numeric and factorial dependent variables.
Step 3. Key parameters
With complete data, the general modeling set was from stratifying random-split cross validation into training data (70% data) and testing data (30% data), containing proportional positive and negative cases, respectively.
    Step 3.1. Parameter composition
    Parameters (e.g., gamma, nu, cost, degree, coef0) optimized separately: their value ranges were determined by the best outputs.
    Parameters' best composition (e.g., gamma, nu, cost): parameters were set by training data through 10-fold 3-time cross validation. Accuracy (total precise rate), F1 score, kappa (consistence), and sensitivity (positive precise rate) values were selected as evaluation indicators.
    Parameter value determination (e.g., gamma, nu, cost): gamma and cost were set as the minimal values; nu was set as the mean value in parameter composition.
    Step 3.2. Regressions for selected parameters
    Regression analysis of parameters (gamma, nu) and corresponding case number were tested for computable correlations.
Step 4. Model prediction performance
The model prediction was performed on testing data and other testing drugs. Four indexes (accuracy, F1, kappa, and sensitivity) and ROC were checked for its effect.

### 2.3. Statistical Analysis

Descriptive analysis was used to summarize patient demographic characteristics, with mean values for continuous variables and ratios for categorical variables. To explain the impacting factors in hyperglycemia, “Reaction” is defined as a dependent variable and others as response variables. *T*-test was performed for comparing normal distributions and defining 95% confidence intervals, and Wilcoxon rank test was used for comparing other unknown distributions. *R* language (version 4.2.0 for Windows) was used for statistics, and its library of e1071 was used for SVM model buildup.

## 3. Results

A demographic summary of complete data for analysis is provided in Table 1. Due to the limited number (only 1) of positive cases in the complete data, cam and cem were not included in model setup. The two drugs as well as ipi were set as testing drugs.

Pilot assay was used for algorithm selection based on proportional 600 cases of each drug. Positive and negative cases were classified as number type (“1,” “0”) or factor type (“Yes,” “No”). Optimization methods were combined as number and R-tune. Accuracy (total precise rate), F1 score, kappa (consistence), and sensitivity (positive precise rate or recall) values were evaluated as indicators of performance. Confusion matrix was calculated according to Table2. Compositions of “fn” and “nn” in complete data displayed best performances in Figure 2.

One key to constructing an SVM model that can accurately screen the active markers is to select the appropriate variable indexes [23]. Classical variable selection methods were near zero variance method and model assessment. Three variables (Nos. 9–11, Table 3) as well as “ID” and “Outcomes” were deleted in the following analysis. “Source” and “Reporter” introduced where the ADR came from, without more clinical information in ADR control; “Outcomes” did not influence “Reactions.” The other 8 variables (Nos. 1–8, Table 3) were selected for model setup.

SVM model is determined by its kernel (“*l*,” “*p*,” “*r*,” “*s*”) and type (“*C*,” “one,” “eps,” “nu”). The five PD-1/L1 drugs were test by the 4 × 4 kernel-type cross compositions. As the index range span is too long, *y*-axis values were logged in the boxplots. In number type, “r-nu” (“rbf” and “nu-regression”) displayed better performances, especially at the important indexes of F1 score and kappa. In factor type, “*p*-*C*” displayed better performances, except for being lower at sensitivity. Moreover, “*r*-nu” performed better than “*p*-*C*” at F1 score and kappa (Figure 3).

As “eps” and “nu” regression need numeric dependent variables, “*r*-nu” and number type/number optimization were selected for SVM model setup.

Generally, modeling set was from stratifying random-split cross validation into training data (70% data) and testing data (30% data), containing proportional positive and negative cases, respectively.

Parameters of SVM mainly included degree, cost, gamma, nu, coef0. From pilot study, nu was defined by the mean value and cost (=1) and gamma by the minimal value in the best prediction range (1∼10); while other parameters did not need to be adjusted. The main model setup algorithm is shown in Algorithm 1.

Main model setup indicated the critical points depended on the patterns of nu and gamma. In regression analysis, we found out that the nu values (0 < nu ≤ 1) were exponential and gamma values (1 ≤ gamma ≤ 10) were quadratic to case number, regression formula, and curves as in (1) and (2) and Figure 4.

(1) $$\begin{array}{c} y=0.5649\times e^{\left(-x/6984\right)}.\left(y=nu,x=\text{case}\right), \end{array}$$

(2) $$\begin{array}{c} y=9.005\times 10^{-4}x-4.877\times 10^{-8}x^{2}.\left(y=\text{gamma},x=\text{case}\right). \end{array}$$

The setup model with optimized parameters (type: nu-regression; kernel: rbf; parameter: nu and gamma from formulas (1) and (2)) was applied on testing-part (5 testing data and 3 drugs). Three indexes (accuracy, F1 score, and kappa) were greatly improved in model than in initial prediction (Figure 5).

Receiver operating characteristic (ROC) analysis was used to describe the discrimination accuracy of a diagnostic test or prediction model [24]. The diagnostic values from this model prediction and single variables (“Reactions,” “Reason,” “Country,” “Weight,” “Year,” “Age,” “Priority,” and “Sex”) on the testing parts were evaluated by ROC curves, whereas the predictive performances were much better from model than single variables in Figure 6.

## 4. Discussion

The application of machine learning in healthcare delivery presents unique challenges that require data preprocessing, model training, and refinement of the system with respect to the actual clinical problem [20]. In this study, we have developed a machine learning algorithm with correct cores and computable parameters.

Hyperglycemia is a serious ADR in cancer treatment [25], and it is urgent to predict occurrence among cancer patients. Hyperglycemia influences the outcome of cancer therapy via various mechanisms such as inflammation sponsoring [1], immune destruction [26]. In inclusion criteria, “Diabetic” is set as an item to include diabetic complications such as ketoacidosis and coma. As PD-1 joint therapies (e.g., nivo combined with ipi, and pem combined with chemotherapy [27]) have been approved by the FDA, ipi is also included for better testing hyperglycemic ADR prediction in drug usage. To the best of our knowledge, this is the first time that hyperglycemia is predicted from real-world clinical practice via machine learning model.

SVM is a kind of structural dependence model to find maximum margin hyperplane with ADR and reported features. To train the algorithm, new cases are projected in the same situation to test which side of the hyperplane they are located on [22]. As the adverse events may have occurred in a small fraction of patients, for class-imbalance, data were split into proportional and random training, and testing parts were performed by *R* library: createDataPartition. SVM is powerful in data mining for better classification; however, it is greatly influenced by the parameters. It is inefficient to use traditional grid search, learning curve, and other parameter adjustment methods [28]. SVM is usually used as control algorithm in diabetic prediction [29], while our model has obtained the optimal parameters effectively considering the key parameters as well as their large space and enhanced the prediction precision, where we discussed its parameter tuning and provided a new conception of parameter adjustment.

In raw data, the high-performance accuracy was from the data itself, as the low hyperglycemic incidence and high negative-case number pushed up its accuracy. In complete data, number optimization performed better than *R*-tune optimization, in that *R*-tune leans toward various minor compositions other than the comprehensive adjustment in number optimization (Figure 2).

Variable selection depended on both statistical and clinical significance. Due to omission values and duplicated cases, variables should be filtered in machine learning. Variable importance was tested by two methods: in near zero variance method, variables displayed “*T*” as deletable; in overall value of model assessment, variables displayed “0” as deletable. Compared the two methods and considered clinical implications, variables of “reactions,” “reason,” “country,” “age,” “weight,” and “year” are included. Though “Sex” is deletable in overall method, “nzv” method indicated it as meaningful. Furthermore, “Sex” was an important parameter clinically, so it was included in variables. For the clinical and algorithmic assessment, “Serious,” “Source,” and “Reporter” were not included in model setup (Table 3).

SVM model is usually based on kernel and type kinds. From crossing composition, “*r*-nu” in number type showed better value than average in accuracy and sensitivity, and top values in F1 score and kappa, and it is better than “*p*-*C*” of factor type (Figure 3). Furthermore, “eps” and “nu” regression did not accept factorial variables. The number type/number optimization and kernel and type of “*r*-nu” composition were selected for SVM model setup. Since SVM-Type of nu-classification did not work in both factor and number here, it was not checked in type and kernel (Step 2.3).

Five parameters (degree, cost, gamma, nu, and coef0) were adjusted in parameter selection (Step 3.1). As no results changed in regulating degree and coef0, the two parameters were set as the function default. To avoid overfitting, cost value was defined as “1” (the function default number). Adjusting the other two parameters (nu and gamma) could improve model performance in 3 × 10 (10-fold 3-time) cross validation. Then, nu was defined by the mean value and gamma by the minimal value from model. Because the whole range of nu (0∼1) had been checked in cross validation, its mean value could cover entire situations. However, gamma determines distribution of new feature space, meaning that the smaller the gamma value, the more the support vectors. So, the choice of gamma on smallest value would not be effected by its primeval testing range. Different from previously published preprint [30], model results from 5 drugs were included because of imported new cases and new positive case criteria. In regression test, we found that if nu was chosen after minimizing gamma value, the prediction performances were not well either at small or big case volume (in linear, partially linear, or nonlinear regression). For balance, we chose gamma from 1∼10, while we chose nu from 0∼1 in this study; Figure 5 displays their good prediction performances.

In the exponential curves (1), the constant value (6984) was iterated from more and more narrow ranges in linear regression between nu value and *e*^(−case number/constant)^(iterated highest *r*^2^).

The positive hyperglycemic ADR case ratio is relatively low (<5%, Table 1), so the mass of negative cases pushed up sensitivity values in initial prediction (Figure 5). The other three indexes could also support this model's good performance. The graphical ROC curve is produced by plotting sensitivity (true positive rate) on the *y*-axis against 1–specificity (false positive rate) on the *x*-axis for the various values tabulated [31]. Areas under the ROC curves (AUC) from single variables were far less than those from model prediction (the uppermost red line in Figure 6). The prediction of composite variable was powerful, since that of every single item is close to the diagonal line separately. In cam and cem, low positive case (only 1 case) influenced single variable prediction, but they were also lower than model prediction (the uppermost red line in Figure 6).

One SVM's downside is that finding the best model requires testing of various compositions of kernels and model parameters. The success or failure of machine learning approaches on a given problem may vary strongly with the expertise of the user [14]. Our model process set up an efficient kernel and composite parameter and improved the prediction for positive cases.

Though SVMs are extremely powerful classifiers and there are no medicolegal implications, clinicians' understanding, or privacy and security on public database, several limitations must be addressed. One thing that needs to be clear is that pharmacovigilance databases can just be used to predict correlations rather than causality. FAERS (including spontaneous reporting systems) declares no certainty that the reported event was due to the product, insufficient details, incomplete reports, and duplicate reports [13]. Other drug factors (e.g., doses, frequency) and biological factors (e.g., genomic data, personal habits) were not included in the development of the present algorithm, which might prevent accuracy and F1 score from rising up to 100%. It should be clear from the narrative examples used in this paper that choice, tuning, and diagnosis of machine learning applications are far from mechanical [32]. Furthermore, (1) and (2) could only function in given case range; if the case number is too huge or small, the model should be re-set up.

Despite the limitations described above, this algorithm has provided meaningful information in order to adjust care goals for these patients or provide signs for further well-organized clinical studies.

ADR is one of the pharmacovigilance keys during drug post-marketing phase. On the one hand, it is challengeable to find out the effective and fast means from clinical heterogeneity results. On the other hand, interestingly, ADR prediction is more important in that its occurrence is usually unknown in clinical treatment, since real time monitoring is expensive and inconvenient for discovering ADRs. This algorithm model from clinical available features at the time of presentation was proved robust and generalizable in later testing-part sequence. This noninvasive and precise prediction could greatly help clinical practitioners to distinguish high-risk patients. Therefore, this study provided an orientation to predict hyperglycemic ADR with these drugs.

## 5. Conclusion

In summary, the SVM model established here can noninvasively and precisely predict hyperglycemic ADR in patients treated with PD-1/PD-L1 inhibitors from given personal-related features and given case number. An SVM model was set up based on compositions of correct kernels and computable parameters. The SVM model showed good prediction performance in testing data, which proved that this model is robust and generalizable in this field. This model setup process provided an analytic conception for promotion to other ADR prediction. We also believe that the availability of medical and personal information will further facilitate this model. Such information from prediction is vital for preventing or even overcoming ADR and to improve patient outcomes by distinguishing high hyperglycemia-risk patients, and this machine learning algorithm can eventually add value to clinical decision making.

## Figures and Tables

**Figure 1:** Flow chart of study process. Step 1: original data fixed into raw data and complete data. Step 2: core SVM algorithm selection. Step 3: adjustment of parameters in 70% complete data to set up model using 3 × 10 cross validation and parameter composition. Analysis optimizing parameters (gamma and nu values) in curve regression. Step 4: model prediction performances in four indexes and ROC curves.

**Figure 2:** Performance for data version and algorithm classification. In raw data: *f*_raw: factor type; *n*_raw: number type. In complete data: nn: number type, number optimization; ft: factor type, *R*-tune optimization; fn: factor type, number optimization. To compare the effect of missing values, raw data and complete data (filtered from raw data) were both checked in the pilot test. The positive cases were marked in the form of factor type (“yes” and “no”) or number type (“1” and “0”); the optimization methods were number and tune. According to SVM model options, there were 5 compositing types. The assessing indexes of tested drugs were checked for the more optimized algorithm. All four indexes in raw data displayed lower scores, while these in algorithms (fn, nn) of complete data displayed highest scores. (a) Accuracy. (b) F1 score. (c) Kappa. (d) Sensitivity.

**Figure 3:** Performance of kernel and type compositions. SVM algorithm is based on its kernel (“*l*,” “*p*,” “*r*,” “*s*”) and type (“*C*,” “one,” “eps,” “nu”). Drugs were tested by the 4 × 4 kernel-type cross compositions. In number type, “*r*-nu” (“rbf” and “nu-regression”) displayed highest score in (b) and (c) and were still in the top class in (a) and (d). In factor type, “*p*-*C*” displayed highest scores in (e)–(g) but lower scores in (h). Comprehensively, “*p*-*C*” (the best in factor type) performed weaker than “*r*-nu” (number type). (a) Accuracy (log *Y*). (b) F1 score (log *Y*). (c) Kappa (log *Y*). (d) Sensitivity (log *Y*). (e) Accuracy (log *Y*). (f) F1 score (log *Y*). (g) Kappa (log *Y*). (h) Sensitivity (log *Y*).

**Figure 4:** Curve regressions of gamma and nu values. nu and gamma values were related to case number of drugs. (a) nu value related to exponent of case number linearly (1). (b) Gamma value related to case number in quadratic curve (2).

**Figure 5:** Prediction performance before/after parameter regression. TCN: total case number, PCN: positive case number in tested parts. *a*: accuracy, *f*1: F1 score, *k*: kappa, *s*: sensitivity. Red columns stand for initial prediction before parameter regression; green columns stand for prediction from model. Model set up from 5 drugs, so only testing data were for checking (a∼e); and another 3 drugs for checking (f∼h). This model improved greatly at indexes of accuracy, F1 score, and kappa, as red column scores were much lower than those of green ones. (a) Avel (test part). (b) Dur (test part). (c) Atez (test part). (d) Pem (test part). (e) Nivo (test part). (f) Ipi. (g) Cem. (h) Cam.

**Figure 6:** Predictive evaluations in terms of ROC curves. in ROC curves, prediction from single items (“reactions,” “reason,” “country,” “weight,” “year,” “age,” “priority” and “sex”) “stay” around diagonal with low area under curve (AUC), while prediction from model (red line) nearly at top in (a∼f). In (g∼h), the single variable did not “stay” around diagonal, maybe because of the influence by limited positive case (only 1); but red lines were still at the top. The predictive performances were much better improved from this model than any single variables. (a) Avel (test part). (b) Dur (test part). (c) Atez (test part). (d) Pem (test part). (e) Nivo (test part). (f) Ipi. (g) Cem. (h) Cam.

**Algorithm 1:** Key model setup algorithm.

**Table 1:** Main characteristics of cases in complete data.

Drugs	TCN (PCN)	PCN (%)	Age (year)	Male (%)	Weight (kg)	Year range
Cam	37 (1)	2.7	55.6 ± 13.2	64.9	59.5 ± 12.4	2017–2021
Cem	52 (1)	1.9	73 ± 13	82.7	76.9 ± 15.8	2018–2021
Avel	1074 (22)	2	65.1 ± 11.6	61.6	75.3 ± 20.8	2014–2021
^*∗*^Dur	1715 (46)	2.7	65.9 ± 10.3	67.6	69.7 ± 18.1	2011–2021
Atez	7073 (133)	1.9	64.2 ± 11.6	56	70.5 ± 18.4	2012–2021
^*∗*^Pem	9416 (310)	3.3	65.8 ± 11.5	63	68.6 ± 20.7	2000–2021
^*∗*^Nivo	15629 (708)	4.5	63.3 ± 12.8	64.3	73.7 ± 22.1	2010–2021
Ipi	7907 (378)	4.8	61.7 ± 13	63.7	77.3 ± 21.4	2007–2021

TCN: total case number. PCN: positive case number. ^*∗*^Cases reported with wrong year were deleted: dur (1979), pem (1921), nivo (2022).

**Table 2:** Confusion matrix and index formula.

	Real *Y*		Real *N*
Predicted *Y*	True positive (TP)		False positive (FP)
Predicted *N*	False negative (FN)		True negative (TN)

Index		Formula		

Precision		(TP)/(TP+FP)		
Accuracy		(TP+TN)/(TP+FP+FN+TN)		
Sensitivity (recall)		TP/(TP+FN)		
P(e)		((TP+FP)^*∗*^(TP+FN)+(FN+TN)^*∗*^(FP+TN))/(TP+FP+TN+FN)^2^		
Kappa		((accuracy – P(e))/(1 – P(e)))		
F1 score		(2/(1/precision)+(1/sensitivity))		

**Table 3:** Variable selection in two methods.

Drugs		Avel		Dur		Atez		Pem		Nivo	
No.	Variable	nzv	Overall	nzv	Overall	nzv	Overall	nzv	Overall	nzv	Overall
1	Reactions	F	1	F	1	F	1	F	1	F	1
2	Reason	F	0.771	F	0.434	F	0.549	F	0.374	F	0.229
3	Country	F	0.033	F	0.005	F	0.004	F	0.004	F	0.009
4	Age	F	0.007	F	0.004	F	0	F	0	F	0
5	Weight	F	0.007	F	0.013	F	0.002	F	0	F	0.001
6	Sex	F	0	F	0	F	0	F	0	F	0
7	Year	F	0	F	0	F	0	F	0.002	F	0
8	Priority	T	0	F	0	T	0.001	F	0.004	T	0.001
9	Reporter	T	0	F	0	T	0	F	0	F	0
10	Serious	T	0	T	0	T	0	T	0	T	0
11	Source	T	0	T	0	T	0	T	0	T	0

nzv: near zero variance. Overall: overall value of model assessment. T: true. F: false (“T” or “0” means this variable should be deleted in each method).

## Data Availability

The data used to support the findings of this study are available from FAERS public dashboard; and algorithm(s) are available from the corresponding author on reasonable request.

## References

[1] Ramteke P., Deb A., Shepal V., Bhat M. K. (2019). Hyperglycemia associated metabolic and molecular alterations in cancer risk, progression, treatment, and mortality. *Cancers*.

[2] Yang J., Jia B., Qiao Y., Chen W., Qi X. (2016). Variations of blood glucose in cancer patients during chemotherapy. *Nigerian Journal of Clinical Practice*.

[3] Patrinely J. R., Johnson R., Lawless A. R. (2021). Chronic immune-related adverse events following adjuvant anti-PD-1 therapy for high-risk resected melanoma. *JAMA Oncology*.

[4] Silva I. P. D., Lo S., Quek C. (2020). Site-specific response patterns, pseudoprogression, and acquired resistance in patients with melanoma treated with ipilimumab combined with anti-PD-1 therapy. *Cancer*.

[5] Wang Y., Zhou S., Yang F. (2019). Treatment-related adverse events of PD-1 and PD-L1 inhibitors in clinical trials: a systematic review and meta-analysis. *JAMA Oncology*.

[6] Barroso-Sousa R., Barry W. T., Garrido-Castro A. C. (2018). Incidence of endocrine dysfunction following the use of different immune checkpoint inhibitor regimens: a systematic review and meta-analysis. *JAMA Oncology*.

[7] Yang J., Gu Q., Wang W., Chen Z., Li N. (2021). Analysis of hyperglycemic adverse drug Reactions of Nivolumab and Pembrolizumab based on FAERS database. *Chin J Pharmacoepidemiol*.

[8] Yang J., Zhao B., Zhou H., Jia B., Chen L. (2022). Blood glucose related adverse drug reaction of antitumor monoclonal antibodies: a retrospective analysis using Vigibase. *Brazilian Journal of Pharmaceutical Sciences*.

[9] Lee C., An D., Park J. (2016). Hyperglycemic memory in metabolism and cancer. *Hormone Molecular Biology and Clinical Investigation*.

[10] Vasconcelos-dos-Santos A., Queiroz R. M. D., Rodrigues B. D. C., Todeschini A. R., Dias W. B. (2018). Hyperglycemia and aberrant O-GlcNAcylation: contributions to tumor progression. *Journal of Bioenergetics and Biomembranes*.

[11] Yang J., Wang Y., Liu K., Yang W., Zhang J. (2019). Risk factors for doxorubicin-induced serious hyperglycaemia-related adverse drug reactions. *Diabetes Therapy*.

[12] Yang J., Yang J. (2019). Hyperglycemic ADR distribution of doxorubicin from VigiBase. *American Journal of Therapeutics*.

[13] Food&Drug Administration US. https://www.fda.gov/.

[14] Huang S., Cai N., Pacheco P. P., Narrandes S., Wang Y., Xu W. (2018). Applications of support vector machine (SVM) learning in cancer genomics. *Cancer Genomics &amp;amp; Proteomics*.

[15] Zhao M., Hoti K., Wang H., Raghu A., Katabi D. (2021). Assessment of medication self-administration using artificial intelligence. *Nature Medicine*.

[16] Deo R. C. (2015). Machine learning in medicine. *Circulation*.

[17] Lakshmanna K., Khare N. (2016). FDSMO: frequent DNA sequence mining using FBSB and optimization. *International Journal of Intelligent Engineering and Systems*.

[18] Li H., Liu J., Wu K., Yang Z., Liu R. W., Xiong N. (2018). Spatio-temporal vessel trajectory clustering based on data mapping and density. *IEEE Access*.

[19] Bernardini M., Romeo L., Misericordia P., Frontoni E. (2020). Discovering the type 2 diabetes in electronic health records using the sparse balanced support vector machine. *IEEE journal of biomedical and health informatics*.

[20] Ngiam K. Y., Khor I. W. (2019). Big data and machine learning algorithms for health-care delivery. *The Lancet Oncology*.

[21] Wang M., Pang Z., Wang Y. (2021). An immune model to predict prognosis of breast cancer patients receiving neoadjuvant chemotherapy based on support vector machine. *Frontiers Oncology*.

[22] Zhang J., Han X., Zhao H. (2018). Personalized prediction model for seizure-free epilepsy with levetiracetam therapy: a retrospective data analysis using support vector machine. *British Journal of Clinical Pharmacology*.

[23] Li S., Wang L., Du Z. (2019). Identification of the lipid-lowering component of triterpenes from Alismatis rhizoma based on the MRM-based characteristic chemical profiles and support vector machine model. *Analytical and Bioanalytical Chemistry*.

[24] Obuchowski N. A., Bullen J. A. (2018). Receiver operating characteristic (ROC) curves: review of methods with applications in diagnostic medicine. *Physics in Medicine and Biology*.

[25] Yang J., Jia B., Yan J., He J. (2017). Glycaemic adverse drug reactions from anti-neoplastics used in treating pancreatic cancer. *Nigerian Journal of Clinical Practice*.

[26] Li L., Chen Y., Chenzhao C., Fu S., Xu Q., Zhao J. (2018). Glucose negatively affects Nrf2/SKN-1-mediated innate immunity in *C. elegans*. *Aging*.

[27] Tang J., Yu J. X., Hubbard-Lucey V. M., Neftelinov S. T., Hodge J. P., Lin Y. (2018). The clinical trial landscape for PD1/PDL1 immune checkpoint inhibitors. *Nature Reviews Drug Discovery*.

[28] Zhang J., Qiu X., Li X., Huang Z., Wu M., Dong Y. (2021). Support vector machine weather prediction technology based on the improved quantum optimization algorithm. *Computational Intelligence and Neuroscience*.

[29] Olisah C. C., Smith L., Smith M. (2022). Diabetes mellitus prediction and diagnosis from a data preprocessing and machine learning perspective. *Computer Methods and Programs in Biomedicine*.

[30] Yang J., Lin W., Shi L., Deng M., Yang W. (2020). A Machine Learning Algorithm to Predict Hyperglycemic Cases Induced by PD-1/PD-L1 Inhibitors in the Real World. *Mapping Intimacies*.

[31] Hoo Z. H., Candlish J., Teare D. (2017). What is an ROC curve?. *Emergency Medicine Journal*.

[32] Tarca A. L., Carey V. J., Chen X. W., Romero R., Draghici S. (2007). Machine learning and its applications to biology. *PLoS Computational Biology*.

